The article "Pesticide Residues and Effect of Household Processing in Commonly Consumed Vegetables in Jimma Zone, Southwest Ethiopia" was published in 2023. Journal: J Environ Public Health.

# Pesticide Residues and Effect of Household Processing in Commonly Consumed Vegetables in Jimma Zone, Southwest Ethiopia

**DOI:** 10.1155/2023/7503426

**Published:** 2023-01-30

**Authors:** Amare Terfe, Seblework Mekonen, Temima Jemal

**Affiliations:** ^1^Department of Environmental Health Science, College of Medicine and Health Sciences, Arba Minch University, P.O.Box 21, Arba Minch, Ethiopia; ^2^Ethiopian Institute of Water Resources, Water and Health, Addis Ababa University, Addis Ababa, Addis Ababa, Ethiopia; ^3^Department of Environmental Health Science and Technology, Institute of Health, Jimma University, P.O. Box 378, Jimma, Ethiopia

## Abstract

The long-term and indiscriminate use of pesticides has resulted in serious health effects. Aside from that, developing countries do not have any monitoring systems in place to prevent the consumption of high levels of pesticides in foods. Therefore, this study aimed to determine pesticide residues and the effect of processing in commonly consumed vegetables in the southwestern part of Ethiopia. In total, 12 samples of 1 kg of each type of vegetable were collected from selected markets. Moreover, as a solution to pesticide residue problems in vegetables, the effect of different processing methods such as washing, peeling, boiling, and their cumulative effect was studied. In the analytical procedure, the modified Quick, Easy, Cheap, Effective, Rugged, and Safe (QuEChERS) extraction with florisil as a cleanup sorbent was used and the identification of pesticides was done by using gas chromatography with an electron capture detector (GC-ECD). The parent *p,p'*-DDT was detected at a concentration of 0.015 mg/kg in potato samples from the Serbo market and a concentration of 0.516, 0.232, 0.174, and 1.512 mg/kg in Merkato, Kochi, Serbo, and Shebe onion samples, respectively. P*`p*-DDT is detected at a high concentration compared to its metabolites *(p,p'*-DDE and *p,p'*-DDD), which is an indication of recent use. DDT and its metabolites, other organochlorines (lindane, *γ*-chlordane, dimethachlor, and heptachlor), and pyrethroids (cypermethrin and deltamethrin) exceeded the recommended limits by FAO and WHO in multiple samples of potato, onion, and cabbage. The processing result showed that washing, boiling, and the combination of the two revealed a 100% reduction in *o,p'*-DDT, and *p,p'*-DDT pesticides detected in cabbage. In conclusion, multiple residues were detected in the three vegetables studied, indicating that pesticides were applied intensively. Pesticide levels were reduced by home processing procedures, which is important for consumer safety.

## 1. Introduction

Worldwide, pesticides have been used in agriculture, horticulture, and public health for the control of pests and disease vectors [1]. Consequently, different pesticides have been applied in agriculture since they are very much effective in avoiding pests and sustaining the quality and quantity of crops. However, those pesticides must be applied according to the recommended guidelines, which consider the type of pesticide used, as well as the dose and intervals at which they are applied [2]. Even though pesticides have improved the standard of human life by controlling pests and vectors, their long-term and indiscriminate use have resulted in serious health effects. As pesticide use has increased over the past few decades, the likelihood of exposure to these chemicals has also increased considerably [3]. Increased use of pesticides is not the only problem; rather, there has been overdosage as well as mixing of different types of pesticides with the assumption of increasing their efficacy in pest control and improving productivity [4]. Despite their inevitable use, pesticides have adverse health effects for consumers because of their residues found in different food items. As a result, food safety is a growing concern worldwide on account of its direct relation to human health [5, 6].

The article "Pesticide Residues and Effect of Household Processing in Commonly Consumed Vegetables in Jimma Zone, Southwest Ethiopia" was published in 2023. Journal: J Environ Public Health.

Furthermore, pest infestation is higher in vegetable crops, which necessitates frequent pesticide application. A high concentration of pesticides in vegetables can be due to the overuse of pesticides. In addition, different types of pesticides might be mixed to increase their efficacy [4, 7]. Among the vegetables that are highly susceptible to pests are onions, potatoes, and cabbage. This could contribute to the successive application and detection of those pesticides at a higher concentration on those vegetables. In vegetable agriculture, pyrethroids and organochlorines were among the commonly detected pesticide residues in different studies [8, 9].

Although developed countries have sophisticated systems already in place to register pesticides, and control their trade and use, this is not always the case in most developing countries [1]. Some existing monitoring programs, mostly in developing countries, are carried out due to the demands of international trade [10]. Therefore, to reduce the risk of exposure to pesticide residues from the consumption of contaminated foods, there has to be a continuous monitoring system for pesticides to prevent those effects. However, that is not the case in most developing countries; even they do not have established maximum residue limits (MRLs) for different pesticides that have been used in the agriculture sector. In addition, those farmers in the developing world lack awareness about the proper dosage, frequency of application, toxicity, and many other issues about pesticides [7, 11, 12].

The article "Pesticide Residues and Effect of Household Processing in Commonly Consumed Vegetables in Jimma Zone, Southwest Ethiopia" was published in 2023. Journal: J Environ Public Health.

Therefore, there is a need to regulate pesticide intake for leading a healthy life using other mechanisms than monitoring. Processing of foods can be one mechanism that substantially reduces the residues of pesticides. Several simple, less labor, and cost-effective food processing methods such as washing, peeling, and cooking singly or in combination can be applied as an effective means of reducing dietary consumption of pesticide residues [13]. Moreover, the reduction of pesticides through processing is essential in decreasing the risk associated with the ingestion of pesticide residues, especially in vegetables [14]. Despite the knowledge gap on the exact mechanism of action of different processing techniques, some processes may lead to an increase in the residue level due to the concentration effect. Thus, there is an increasing need for information about the effects of various processes on the fate of pesticide residues in foods from a public health concern perspective [15].

Despite the presence of pesticide contamination, the Ethiopian population continued living by consuming those risky foods. Different studies in Ethiopia showed that food products are contaminated with pesticides and banned pesticides are still being used illegally in the agricultural sector. However, still Ethiopia did not have a pesticide monitoring system for those pesticides in food products [7, 11]. However, different studies showed that food processing has a significant impact on reducing the levels of pesticides in cereal foods [14, 16, 17]. Traditionally, different processing techniques like washing, peeling, boiling, and their combinations have been practiced in Ethiopia for different types of foods including vegetables. Therefore, this study aimed to determine the level of pesticides and the effect of household processing on commonly consumed vegetables in Ethiopia.

## 2. Materials and Methods

### 2.1. Study Area and Design

The study was conducted in purposively selected urban markets in the Jimma zone, southwest Ethiopia, which are known as a source of vegetable supply for the community. Four major marketplaces were included in this study (Merkato and Kochi markets from Jimma town, Shebe market from Shebe woreda, and Serbo market from Kersa woreda). A laboratory-based cross-sectional study design was conducted in the Jimma zone, southwest Ethiopia, from June 1 to July 28, 2021. The study area was indicated in the map below (Figure 1).

### 2.2. Sample Collection

A total of 12 vegetable subsamples for each vegetable type were collected from four urban vegetable markets selected for this study (3 subsamples from each market for each vegetable). About 36 vegetable samples were collected from four marketplaces. Moreover, the vegetables were purchased from sellers who sell vegetables by purchasing from multiple farmers to increase the representativeness of the sample. A 1 Kg or 10 units (heads) of each commonly consumed vegetable in the Jimma zone was purchased from those purposively selected four markets. This study had four samples, each with three subsamples to make composite samples of each vegetable for one sampling point. After purchasing the three subsamples from one market for each vegetable under this study, the vegetables were separately sealed with aluminum foil, labeled, and then transported to Jimma University Environmental Laboratory for further laboratory analysis. The samples were refrigerated at 4°C before sample extraction and cleanup processes.

The article "Pesticide Residues and Effect of Household Processing in Commonly Consumed Vegetables in Jimma Zone, Southwest Ethiopia" was published in 2023. Journal: J Environ Public Health.

### 2.3. Chemicals and Reagents

The chemicals and reagents used for this study were as follows: analytical grade n-hexane, acetone, acetonitrile, methanol, glacial acetic acid, and for cleanup purposes, anhydrous magnesium sulfate, sodium acetate, and florisil, and for centrifugation, 50 ml and 15 ml centrifuge tubes were used. Commonly studied pesticides by different scholars in Ethiopia were used to be studied in this study, which include *o,p'*-DDT, *p,p'*-DDT, *p,p'*-DDE, *p,p'*-DDD, cypermethrin, and deltamethrin, which were identified from different food matrices and water by [11, 18, 19] and expected to be detected in commonly consumed vegetables. In addition, other pesticides were selected based on the availability of their standards. Therefore, eight organochlorine pesticides and metabolites including *o,p'*-DDT, *p,p'*-DDT, *p,p'*-DDE, *p,p'*-DDD, *γ*-chlordane, dimethachlor, lindane, and heptachlor and two pyrethroids (cypermethrin and deltamethrin) were selected for this study. The analytical purity of those pesticide standards, extraction solvents, and salts was greater than 98%.

### 2.4. Preparation of Stock, Intermediate, and Working Standard Solutions

Individual stock standard solutions containing 1000 mg/L of each of the eleven pesticides under study were separately prepared by dissolving 50 mg of each pesticide standard in 50-ml volumetric flasks based on the pesticide solvent choices and stored at 4°C. Intermediate solutions of 100 mg/L were prepared by diluting 1 ml of the stock solution with 9 ml of the solvent (methanol or acetone). Finally, working solutions of 0.001, 0.01, 0.1, 1, and 10 mg/L were prepared following serial dilution for each pesticide.

### 2.5. Sample Preparation Procedure

#### 2.5.1. Sample Preparation for Quantification of Pesticides

From every three subsamples, an equal proportion of vegetables were taken to make a composite sample of 1 Kg for one sampling point for each vegetable. 1 Kg of each vegetable was homogenized in a household electric homogenizer/juicing machine to obtain a homogenous matrix. Then, from the homogenized sample, 5 g was taken for extraction and cleanup processes.

The article "Pesticide Residues and Effect of Household Processing in Commonly Consumed Vegetables in Jimma Zone, Southwest Ethiopia" was published in 2023. Journal: J Environ Public Health.

#### 2.5.2. Sample Preparation for Processing

A mixture of eleven pesticide standards was selected to be studied with 500 *μ*l of each pesticide containing a concentration of 1 mg/L spiked on the surface of the potato, onion, and cabbage samples. The spiked vegetable samples were dried in the open air at room temperature for 30 minutes and then refrigerated at 4°C for 24 hours before the extraction and cleanup process as applied by [20, 21] with slight modification. Those spiked vegetable samples were processed according to the methods for determining the effect of different household processing methods on pesticide residues in commonly consumed vegetables, in southwest Ethiopia.

### 2.6. Sample Extraction and Cleanup

According to different studies, the QuEChERS procedure using the acetate-buffered version presented higher and more consistent recoveries for most compounds including pH-dependent pesticides [22–24]. Therefore, to determine the level of pesticides in the vegetables under study, the acetate-buffered QuEChERS sample extraction procedure as used in [22, 25] and dispersive solid phase extraction (d-SPE) cleanup technique with anhydrous MgSO_4_ and florisil according to [25] was applied in this study with slight modifications in the amount of the solvent, cleanup, and extraction chemicals used. Generally, the QuEChERS extraction and cleanup method was used in different studies to analyze pesticide residues in vegetables with high water content. The extraction process was conducted with the following procedures: 5 g of homogenized vegetable as used by [26] was weighed on analytical balance carefully and transferred into a 50-ml centrifuge tube; then, 15 ml of acetonitrile mixed with 1% glacial acetic acid was added to each vegetable sample and the mixture was vigorously shaken by hand for 1 min. 2 g of anhydrous MgSO4 and 1 g of sodium acetate were added into the mixture, shaken by hand for 1 min, and centrifuged at 4000 rpm for 5 min. Then, 2 ml of the supernatant/organic layer containing the solvent and the extracted pesticides was transferred into a 15-ml centrifuge tube containing 300 mg anhydrous MgSO_4_ and 400 mg florisil for cleanup. Again, the tube was shaken for 1 min by hand and centrifuged at 4000 rpm for 5 min. 1 ml of the supernatant was transferred into a 250-ml volumetric flask and evaporated using a rotary evaporator at 40°C and concentrated. Then, 2 ml of n-hexane was added to the flask for reconstituting/solvent exchange purposes. Finally, 1.5 ml was transferred from the flask into 1.5-ml vials for GC-ECD analysis.

The article "Pesticide Residues and Effect of Household Processing in Commonly Consumed Vegetables in Jimma Zone, Southwest Ethiopia" was published in 2023. Journal: J Environ Public Health.

### 2.7. Laboratory Procedures for the Determination of the Effect of Processing on Pesticide Residues

Commonly consumed vegetables selected to be studied in this study undergo various vegetable processing techniques were applied as mentioned by [27] and using local household processing methods in Ethiopia for potatoes, onions, and cabbage. The household processing methods were applied as follows:

#### 2.7.1. Washing

Washing is an important step normally carried out after removing dirt from the harvest of vegetables. The washing process in this study was done using tap water, which resembled the traditional washing process for vegetables in most households in Ethiopia. In the washing process, approximately 250 g of spiked vegetable samples was washed with running tap water by hand rubbing for 2 minutes according to a study done by [28, 29], and soaked in 500 ml of water for 3 minutes at room temperature (25–30°C) [30, 31] with slight modifications in time used for washing and soaking. After the soaking process, the vegetables were separated from the water used for soaking and became ready for the extraction and cleanup process.

#### 2.7.2. Peeling

The peeling process was done mechanically with a knife, which will remove those unwanted or inedible parts of vegetables, mainly the skin. In this study, only a knife was used to remove the skin of potatoes up to 1–1.5 mm of the skin as applied by [29], whereas in onion, 2 to 3 layers of onion were removed until the nonedible part was removed. However, peeling was not applied to cabbage since it is not practiced in household processing in Ethiopia.

#### 2.7.3. Boiling/Cooking

The boiling/cooking process in this study involved immersing the vegetables in 500 ml of boiling water as indicated by [28, 29] until they are cooked, which was checked by the softness of the vegetables when pierced with a knife, which is a common method that is used in home processing of most vegetables in Ethiopia, particularly potato. In this study, the boiling of onion and cabbage was checked visually to determine whether they are cooked or not to resemble the traditional methods in almost all Ethiopian households. Moreover, for cabbage, boiling was also applied by taking 250 g of cabbage boiled in 500 ml of water on a local stove for 30 minutes as well as 1 hour to see the difference with the local method.

#### 2.7.4. Combined Processing Procedures

Washing + peeling + boiling: approximately 250 g of pesticide spiked vegetable samples was first washed by a hand rubbed under running tap water for 2 minutes and then soaked for 3 minutes followed by peeling the outer layer up to the nonedible part, which was removed. Then, the peeled vegetables were boiled in an open boiling system with a more than 1-liter capacity beaker containing 500 ml water until soft (10–15 minutes) for potatoes but checked visually for onions. For cabbage, approximately 250 g of pesticide spiked cabbage samples was first washed by hand rubbing under running tap water for 2 minutes and then soaked for 3 minutes, followed by boiling in an open boiling system with more than 1-liter capacity beaker containing 500 ml water. Whether the cabbage is boiled enough or not was checked visually, which is a common procedure in Ethiopian households. Moreover, the same 250 g of cabbage sample, which underwent the washing process, was also boiled for 30 minutes as well as 1 hour in an open boiling system with a more than 1-liter capacity beaker containing 500 ml water.

The article "Pesticide Residues and Effect of Household Processing in Commonly Consumed Vegetables in Jimma Zone, Southwest Ethiopia" was published in 2023. Journal: J Environ Public Health.

### 2.8. Determination of the Processing Factor (PF)

The processing factor is the proportional amount by which pesticide residues change when food is processed. The processing factor in this study was determined according to the study done by [32].

The processing factor was calculated based on the following formula:

(1) $$\begin{array}{c} Processing\;factor=\frac{Mean\;concentration\;of\;pesticide\;residues\;in\;vegetables\;after\;processing}{Mean\;concentration\;of\;pesticide\;residues\;in\;vegetables\;before\;processing}. \end{array}$$

Finally, after obtaining the processing factor, the percent reduction was calculated by using the following formula: % reduction = (1 − PF) × 100.

### 2.9. Pesticide Identification and Quantification

All pesticide residue identification and quantification were performed using Agilent Technologies 7890A Gas-Chromatography with Electron Capture Detector (GC-ECD) with an ALS auto-sampler for both organochlorine and pyrethroid pesticides. The instrument condition was set by following [16] procedure for the determination of organochlorine and pyrethroid pesticides with slight modifications like using nitrogen gas as a carrier instead of helium gas. A column of 30 m × 3.20 mm internal diameter and 0.25 *μ*m film thicknesses were used with the following oven temperature program: an initial temperature of 80°C, ramped at 30°C min^−1^ to 180°C, ramped at 3°C min^−1^ to 205°C, held for 4 min, ramped at 20°C min-1 to 290°C, held for 8 min. The total GC run time was 27.92 min. Nitrogen was used as a carrier gas at a flow rate of 45 mL min^−1^ and a pressure of 10.04 psi. A *μ*ECD detector was used at a temperature of 300°C using nitrogen as a makeup gas at a flow rate of 60 mL/min. An aliquot of 1 *μ*L was injected in splitless mode at an injection temperature of 250°C.

The article "Pesticide Residues and Effect of Household Processing in Commonly Consumed Vegetables in Jimma Zone, Southwest Ethiopia" was published in 2023. Journal: J Environ Public Health.

### 2.10. Gram Equivalent Calculation

The gram equivalent of the sample (mg/ml) extract was calculated by a formula used according to [11] since we used a solid food matrix, which requires changing the mg/l result into mg/g or mg/kg.

(2) $$\begin{array}{c} Y=A/B*X/Z, \end{array}$$

where *Y*  is gram sample equivalent/ml of extract.

 
*A* = gram of sample extracted
 
*B* = ml of solvent added for extraction
 
*X* = ml of extract taken to the vial for analysis
 
*Z* = ml of n-hexane solvent used for the final reconstitution

### 2.11. Quality Control

An analytical method that was already validated by different scholars [25, 26, 33] with its effectiveness in determining organochlorine, as well as pyrethroid pesticide residues using GC-ECD for quantification, was used in this study. LOD was calculated as three times higher than the level of noise, and the LOQ was equal to ten times the noise level. The validated method we used was with % recovery in the range of 84 to 117% (between 70 and 120%), and limit of detection and limit of quantification range from 0.01 to 4 *μ*g/l and 0.06 to 14 *μ*g/l and % RSD range between 1 and 14% (<20%) (Table 1). These all are in the accepted analytical range according to European Document SANTE/12682/2019 (Directorate General for Health and Consumers, European Union, 2011) [34]. The calibration curve for each pesticide residue was obtained by spiking a mixture of those pesticide standards under study using five concentrations ranging from 0.001 up to 10 mg/L. The linearity was determined by using the coefficient of determination (*r*^2^) from the calibration curve. The coefficients of determination (*r*^2^) for the ten pesticides under study were greater than 0.997. The quantification and identification of pesticide residues were done based on the retention time and peak areas for each pesticide residue. The extraction was done in triplicate for the determination of pesticide residue from the four sampling points for each vegetable, and the mean concentration was computed accordingly.

### 2.12. Statistical Analysis

The data from the GC-ECD were printed and entered into an excel sheet for calculating pesticide concentration using the equation of calibration curves. All pesticide quantification processes were done in triplicate and presented as mean ± standard deviation. The pesticide concentration data were entered into SPSS version 20 for further analysis. One-way ANOVA parametric test was used for pesticide residues with normally distributed data, and Kruskal–Wallis nonparametric test at *P* < 0.05 with *α* = 0.05 was used for pesticide residues without normally distributed data to see the presence of significant difference among the effects of different processing techniques. For the ANOVA test, Tukey's multiple comparisons were used to determine the interaction between those household processing techniques. Shapiro–Wilk normality test was used to check the normality of the data at *P* < 0.05.

The article "Pesticide Residues and Effect of Household Processing in Commonly Consumed Vegetables in Jimma Zone, Southwest Ethiopia" was published in 2023. Journal: J Environ Public Health.

## 3. Results

### 3.1. Pesticide Residues in Commonly Consumed Vegetables

From the ten pesticides studied, six pesticide residues (cypermethrin, deltamethrin, heptachlor, *γ*-chlordane, lindane, and dimethachlor) were detected in potatoes in each of the four sampling points. A potato sample from the Serbo market had the highest mean concentration of 6.31 mg/kg for cypermethrin residue, while potato samples collected from the Merkato market had the lowest mean concentration (0.003 mg/kg) for *p,p'*-DDE. Moreover, all pesticide residues were detected in onion from each of the four sampling points. In all sampling points, *p,p'*-DDE was detected at the lowest mean concentration (0.003 and 0.001 mg/kg) in onion samples collected from Kochi and Serbo markets, respectively, compared to other pesticide residues. On the contrary, cypermethrin was detected in onion samples with the highest mean concentration of 47.45, 138.7, 90.35, and 365.08 mg/kg in Merkato, Kochi, Serbo, and Shebe samples, respectively.

In the case of cabbage, six pesticide residues (lindane, heptachlor, *γ*-chlordane, dimethachlor, cypermethrin, and deltamethrin) were detected in each of the four sampling points. Cabbage sample from Merkato had the highest mean concentration of 6.35 mg/kg of dimethachlor, while the lowest mean concentration of lindane (0.003 mg/kg) in Serbo and *γ*-chlordane (0.004 mg/kg) in Merkato samples. However, *o,p'*-DDT, *p,p'*-DDD, *p,p'*-DDE, and *p,p'*-DDT residues were not detected in each of the sampling points (Table 2).

### 3.2. Effect of Processing

In the washing process, the processing factor for *o, p'*-DDT, *p,p'*-DDD, *p,p'*-DDE, *p,p'*-DDT, cypermethrin, and *γ*-chlordane was less than 1 (PF < 1). The washing process concentrated on deltamethrin (PF = 2.02), lindane (PF = 1.56), heptachlor (PF = 1.46), and dimethachlor (PF = 2.25) pesticide residues in potatoes, while only cypermethrin (PF = 11.05) and deltamethrin (PF = 1.42) have been concentrated by the washing process in onion samples. The washing process had a reduction effect on pesticides *o, p'*-DDT, *p,p'*-DDT, and dimethachlor (PF < 1, reduction), respectively, with a processing factor of 0.36, 0, and 0.72 in cabbage (Table 2).

The article "Pesticide Residues and Effect of Household Processing in Commonly Consumed Vegetables in Jimma Zone, Southwest Ethiopia" was published in 2023. Journal: J Environ Public Health.

The processing factor for the peeling process in potatoes was less than 1 for *o, p'*-DDT (PF = 0.35), *p,p'*-DDD (PF = 0.91), *p,p'*-DDE (PF = 0.17), and *γ*-chlordane (PF = 0.75). On the contrary, *o,p'*-DDT, *p,p'*-DDT, cypermethrin, and *γ*-chlordane had a processing factor greater than 1, which are stated as 1.04, 1.18, 9.35, and 1.50, respectively, in the onion sample. From one-way ANOVA test, there was a significant difference in the mean concentration of *p,p'*-DDE (*P*=0.01) between unprocessed and peeled potatoes, which revealed the concentration decreases during processing (Table 1).

Based on the data indicated in Table 1, the boiling process had a processing factor of 0.43, 0.98, 0.91, 0.49, and 0.68 for *o,p'*-DDT, *p,p'*-DDD, *p,p'*-DDE, *p,p'*-DDT, and *γ*-chlordane residues in the potato, which indicates the reduction factors. Only *p,p'*-DDE had a processing factor of 1.23 in the case of onion in the boiling process. From one-way ANOVA result, there is a significant difference (*P*=0.004) in the mean concentration of boiled and unprocessed cabbage for *p,p'*-DDD pesticide residue (Table 2).

A combined process of washing, peeling, and boiling in the case of potatoes indicated that only cypermethrin had a PF score of 2.97 and it is concentrated in potatoes. In the combined processing of onion, all the pesticide residues have a processing factor of less than 1. Besides, from the ANOVA test results for pesticides, the mean concentration of *p,p*'-DDD (*P* = 0.009), *p,p'*-DDE (*P* = 0.005), and *γ*-chlordane (*P* = 0.02) was significantly different between unprocessed potato and using the combined processing method. Moreover, there was also a significant difference in the mean concentration of heptachlor in washing (*P* = 0.003), peeling (*P* = 0.001), boiling (*P* = 0.0001), and combination of the three processes (*P* = 0.0001) compared with the mean concentration of unprocessed onion (Table 3).

## 4. Discussion

The residues of ten pesticides such as *o, p'*-DDT*, p,p'*-DDT, *p,p'*-DDD, *p,p'*-DDE, cypermethrin, deltamethrin, heptachlor, lindane, dimethachlor, and *γ*-chlordane were studied in three commonly consumed vegetables (potato, onion, and cabbage) in southwest Ethiopia. From the studied pesticides, the concentration of lindane (0.02, 0.04, 0.05, and 0.06 mg/kg) in potato samples from all sampling points was above the Codex MRL of 0.01 mg/kg, which indicates the illegal use of this pesticide in the study areas both from recent and historical applications. Similar to this study, the study done in South Africa detected *o, p'*-DDT*, p,p'*-DDE, and *γ*-chlordane levels in potatoes, which were below their respective MRLs. However, the result for heptachlor and lindane pesticide residues in potatoes in the South Africa study was in complete disagreement with this study, which was above their Codex MRLs [35]. In this study, the mean concentration of parent *p,p'*-DDT in potatoes from the Serbo sample was higher than its metabolites (*p,p'*-DDD and *p,p'*-DDE). The detection of the parent *p,p'*-DDT in potatoes above the concentration of its metabolites (*p,p'*-DDD *and p,p'*-DDE) is an indication of the recent use of DDT in potato agriculture in the study areas, which is supported by a study done by [36].

The article "Pesticide Residues and Effect of Household Processing in Commonly Consumed Vegetables in Jimma Zone, Southwest Ethiopia" was published in 2023. Journal: J Environ Public Health.

From the detected DDT metabolites, the concentration of *p, p'*-DDE (0.582 and 0.013 mg/kg) from Merkato and Shebe onion samples exceeded the MRL value of 0.01 mg/kg. The concentration of cypermethrin in all onion samples also exceeded both the Codex and EU MRLs of 0.01 and 0.1 mg/kg, respectively. The residue of Lindane in onion samples also violated the codex MRL of 0.01 mg/kg [37, 38]. A similar finding was reported by [39] in a study done in Ghana, which reported lindane (0.019 mg/kg) and *p,p'*-DDE (0.023 mg/kg) exceeded their respective Codex MRLs in onion. The result of the study in onion showed a higher concentration for cypermethrin and *p,p'*-DDD when compared with the study by [40] in Tanzania, which reported cypermethrin and *p,p'*-DDD had a concentration of 0.014 and 0.01 mg/kg in the onion samples. Moreover, the mean concentration of *p,p'*-DDT and heptachlor pesticide residues in all onion samples was above their DMRL value of 0.01 mg/kg. This result was not comparable with the study in Ghana, where heptachlor and *p,p'*-DDT pesticide residues in all onion samples were below their MRLs [41]. The result could be explained by the lack of awareness of the farmers about the application dose, method of application, and withholding periods.

The mean concentration of DDT and its metabolites *(p,p'*-DDD and *p,p'*-DDE) in potato and onion vegetables are shown in Table 3, and the mean concentration of *p,p'*-DDT was higher than its metabolites in potato samples from Serbo with 0.232 mg/kg and in onion samples of Kochi, Serbo, and Shebe with 0.015, 0.174, and 1.512 mg/kg, respectively. The result was consistent with the study done in the central rift valley of Ethiopia [42], which reported *p,p'*-DDE and *p,p'*-DDT were detected in all samples of onion with a concentration of 0.16 and 0.13 mg/kg, respectively. This is an indication that there might be environmental contaminations from the recent application of DDT in the vegetable areas for control of malaria, which is a common case in Ethiopia [16]. Moreover, the existence of banned organochlorine pesticide residues in onion, potato, and cabbage may be due to their illegal use and their persistence [7, 39].

The article "Pesticide Residues and Effect of Household Processing in Commonly Consumed Vegetables in Jimma Zone, Southwest Ethiopia" was published in 2023. Journal: J Environ Public Health.

DDT isomers (*p,p'*-DDT and *o,p'*-DDT), as well as its metabolites (*p,p'*-DDE and *p,p'*-DDD), were not detected in all cabbage samples. This may be an indication that DDT and its metabolites were not used in cabbage farming from those sampling areas. Apart from that, those pesticides may be below their limit of detection, which is consistent with a study from Ghana [43]. However, the result of this study was against the study done in Senegal and Tanzania, which reported the most critical commodity with multiple existences of pesticides including DDT and its metabolites were cabbage [8, 40].

Cypermethrin pesticide residues in all cabbage samples exceeded the Codex MRL of 0.7 mg/kg with mean concentrations of 2.99, 3.24, 2.87, and 2.79 mg/kg for Merkato, Kochi, Serbo, and Shebe samples, respectively. Similarly, in a study from Tanzania, cypermethrin pesticide residues in cabbage ranged from 2 mg/kg to 3 mg/kg [40]. On the other hand, lindane in Kochi (0.03 mg/kg) and Shebe (0.03 mg/kg) and heptachlor in Shebe (0.25 mg/kg) samples violated their Codex and EU MRL of 0.01 mg/kg [37, 44]. The result for heptachlor pesticide residue (0.017 mg/kg) in the Nigerian study was consistent with this study [45]. However, the result for lindane and heptachlor pesticide residues in cabbage contradicted previous studies [35, 46] in Togo and South Africa, which found that they were detected below their EU MRLs. This discrepancy may be due to Ethiopian farmers overusing pesticides in the hopes of increasing their efficiency.

Regarding multiresidues, there was a coexistence of multiple pesticide residues in commonly consumed vegetables. In onion and potato samples, each sampling point consists of at least seven pesticide residues out of ten pesticides. Similarly, dimethachlor, *γ*-chlordane, lindane, heptachlor, deltamethrin, and cypermethrin were detected at each of the four sampling points in cabbage. The result of this study was in line with the study by [6, 39] stating more than 2 pesticides could co-occur especially in vegetables that are highly pest sensitive. The co-existence of pesticide residues also showed the intensive use of those pesticides in the past as well as in the present [36]. In developing countries, pesticides are not handled and applied according to good agricultural practices to minimize environmental or food commodity contamination [47].

More importantly, this study also examined the percentage reduction of pesticide residues in potato, onion, and cabbage after different processing methods. The results of this study revealed that heptachlor concentrations were significantly different after the washing process (*P*=0.003) in onion, which is consistent with a study by [48] that found heptachlor concentrations were significantly reduced after washing (*P*=0.0018). The present study was in good agreement with the findings found by [49]. They found that washing with water reduced 45% malathion residues from yard-long beans and 41% fenitrothion from eggplant. Moreover, pesticide residues of *o, p'*-DDT (PF = 0.36), *p,p'*-DDT (PF = 0), and dimethachlor (PF = 0.72) were also reduced by the washing process in cabbage. The above result could be explained by the fact that dimethachlor pesticide has the highest water solubility of 2300 mg/l and a low log octanol-water partition coefficient (logP) of 2.17 compared with the other pesticides [50]. This result is consistent with the study by [51] indicating a similar pattern; acetamiprid, with a low log *P*=0.8 and high solubility in water 2950 mg/L, exhibited a low PF = 0.43; in contrast, deltamethrin (log *P*=4.6, water solubility of 0.0002 mg/L) exhibited a PF = 0.73. The result indicated that the logP and solubility were the key factors affecting the reduction of pesticide residues from different food matrices [21]. Moreover, the waxes on vegetable skins also absorb and retain pesticides with high octanol-water partition coefficients, which makes it difficult to remove pesticide residues by washing [52].

The article "Pesticide Residues and Effect of Household Processing in Commonly Consumed Vegetables in Jimma Zone, Southwest Ethiopia" was published in 2023. Journal: J Environ Public Health.

It is also important to keep in mind that different factors such as temperature as well as washing methods have an impact on pesticide residue removal [53]. This study also revealed that low logP and higher water solubility could be the reasons with significant effects on pesticide residues when using washing processing methods to reduce pesticide residues, which complies with the study by [54]. However, high solubility and low logP may not have the same effect on every pesticide residue. When washing potatoes, cypermethrin, a nonsystemic pesticide, was reduced by 17%. This could be due to the mode of action of the pesticides, which plays a significant role in removing pesticide residues [50, 55]. Besides, the result is consistent with the studies done by [14, 51], which indicated washing reduced cypermethrin pesticide residue.

In peeling, the pesticide's mode of action is critical. Systemic pesticides penetrate vegetables, while contact pesticides remain on the skin's surface. Peeling is often associated with nonsystemic pesticides since those pesticides cannot be absorbed by the plant's leaf [29, 56]. This explains the result of this study, which showed that the peeling process caused a processing factor score of less than 1 for five pesticides in potatoes. The reduction was observed in *o,p*'-DDT (65%), *p,p*'-DDD (9%), *p,p*'-DDE (83%), and *γ*-chlordane (25%) in which all of them are nonsystemic pesticides [50], which tend to adhere to the skin of the potato. Those pesticides could be adsorbed to the plant surface resulting in a reduction by the peeling process [57]. Besides, those pesticides also have low water solubility in which they are hardly transported into the internal part of the vegetable [58]. The one-way ANOVA test result also showed that the mean concentration in *p,p*'-DDE(*P*=0.01) is significantly different between unpeeled and peeled potatoes. This is explained by the lipophilic properties of the *p,p'*-DDE with a high logP of 6.51 compared with other pesticides [50, 59].

The article "Pesticide Residues and Effect of Household Processing in Commonly Consumed Vegetables in Jimma Zone, Southwest Ethiopia" was published in 2023. Journal: J Environ Public Health.

On the other hand, pesticide residues of *o, p'*-DDT, *p,p'*-DDT, cypermethrin, and *γ*-chlordane were concentrated in onion resulting in a processing factor of 1.04, 1.118, 9.35, and 1.5 for the peeling process, respectively. This might be due to the nature and composition of the onion such as water content and surface area. Besides, the location of pesticides in different parts of food varies with the nature and type of food commodity and environmental conditions [60]. The results were in line with the study done by [53], which found that residues of the same pesticides can be reduced in different ways on different plants using the same process. In addition, peeling does not always result in pesticide residue reduction due to its systemic action. Pesticide residues are reduced based on the amount of pesticide residue that penetrates the flesh of the processed food to the nature of the processed food commodity [55].

Boiling is the process of cooking food in hot water. In contrast to pesticides with low boiling points, pesticide residues with high boiling points could not be reduced by boiling [29, 61]. In compliance with this fact, cypermethrin, deltamethrin, lindane, heptachlor, and dimethachlor pesticide residues with high boiling points became concentrated in potatoes. On the contrary, *o,p*'-DDT (57%), *p,p*'-DDT (51%), *p,p*'-DDD (2%), *p,p'*-DDE (9%), and *γ*-chlordane (32%) pesticide residues with high boiling points also showed a reduction in concentration from the unprocessed potato. The result could mean that the boiling point is not the only factor in removing pesticide residues; it is also influenced by the amount of time, temperature, moisture loss, and whether the boiling system is closed or open [47].

On the other hand in cabbage, only cypermethrin pesticide residue was concentrated (PF = 2.00), while the other pesticide residues showed a reduction in mean concentration from 5% in heptachlor to 100% in *o, p'*-DDT and *p,p'*-DDT. The result from the boiling process could be due to the boiling point of each pesticide residue, or it could be due to the decomposition by heat or solubility in water [62]. As expected, cypermethrin pesticide residues with high boiling points, hardly soluble in water, thermally stable in heat, and with high log *P*=5.5 [50, 59] became concentrated by the boiling process. The result is similar to the study by [51], which revealed cypermethrin pesticide residue was concentrated (PF = 1.76) by boiling for 5 minutes at 100°C.

The article "Pesticide Residues and Effect of Household Processing in Commonly Consumed Vegetables in Jimma Zone, Southwest Ethiopia" was published in 2023. Journal: J Environ Public Health.

The combined process of washing, peeling, and boiling, which was applied to onion and potato, showed a minimum of 29% reduction in dimethachlor and a maximum of 100% reduction in *o,p'*-DDT pesticide residues in potatoes. But, cypermethrin was highly concentrated in the combined process in potatoes. In the case of onion, the combined process caused a reduction of above 69% in all pesticide residues studied in this study. Physicochemical properties of the pesticides or the vegetable's nature could explain the combined process's outcome in onion and potato [50, 59, 60]. It is more effective because it combines the effects of those three processes, any one of which could contribute to the reduction of pesticide residues.

A local method of washing and soaking for 5 minutes followed by boiling was studied for cabbage. In addition, the cabbage was washed and then boiled for 30 minutes and an hour to compare the time variations with the local visual confirmation method. There was a minimum reduction of 5% in heptachlor up to 100% in *o,p*'-DDT and *p,p'*-DDT pesticide residues using local washing followed by the boiling method. Similar to the local method, washing followed by 30 min boiling in cabbage caused cypermethrin to concentrate. However, it resulted in a minimum reduction of 7% in deltamethrin and a maximum reduction of 100% in *o,p'*-DDT pesticide residues. The finding of this study was against a previous study by [62], which found that washing followed by boiling reduced cypermethrin residue. But, deltamethrin residues were found to be reduced by washing followed by boiling, which is consistent with this study.

## 5. Conclusions

From this study, it appears that there was an intensive use of pesticides in potato, onion, and cabbage cultivation. There was also the co-existence of multiple residues on those vegetable samples from different sampling points. Aside from that, the pesticide concentrations detected in the vegetable samples exceeded the FAO/WHO and EU maximum residue limits (MRLs). Some banned pesticides and those not authorized for use in vegetables such as organochlorines (e.g., DDT, Lindane) were also detected. Recent use of DDT was also observed in the study area. The establishment of MRLs for vegetables and other food products for pesticides used in the cultivation of these crops is necessary to safeguard consumer health in Ethiopia. As a result, there is a need for frequent monitoring of pesticide residues from different food products before they are brought into the market and available for consumption to assure food safety. More importantly, different household processing techniques such as washing, peeling, boiling, and a combination of these processes have a reduction effect on the pesticide residues in the vegetables studied. Even the most persistent organochlorine pesticide residues have been reduced from their original concentration. This is important for the safety of consumers, and it is good to prompt the consumption of vegetables after processing.

The article "Pesticide Residues and Effect of Household Processing in Commonly Consumed Vegetables in Jimma Zone, Southwest Ethiopia" was published in 2023. Journal: J Environ Public Health.

## Figures and Tables

**Figure 1:** Map of the study area.

**Table 1:** Method validation result including recovery, LOD, and LOQ.

Pesticides	% Recovery	% RSD	LOD (*μ*g/l)	LOQ (*μ*g/l)
p,p'-DDE	85	12.3	0.02	0.06
p,p'- DDD	89	13.8	0.02	0.01
o,p'-DDT	95	7.2	0.01	0.04
p,p'-DDT	94.2	1.6	0.02	0.06
ˠ-chlordane	84	12.6	0.03	0.12
Lindane	116	14.4	0.03	0.1
Dimethachlor	86	13.2	0.04	0.14
Heptachlor	92	11.1	0.07	0.22
Cypermethrin	113.5	4.9	4	14
Deltamethrin	117.3	1.3	2	8

**Table 2:** Mean concentration ± SD (mg/kg) of pesticide residues in commonly consumed vegetables in Jimma zone, southwest Ethiopia, 2021.

Pesticide residues	Mean pesticide residue concentration in potato samples				MRL mg/kg	Mean pesticide residue concentrations in onion sample				MRL mg/kg	Mean pesticide residue concentrations in cabbage samples				MRL mg/kg
	S_1_	S_2_	S_3_	S_4_		S_1_	S_2_	S_3_	S_4_		S_1_	S_2_	S_3_	S_4_	
*o,p'*-DDT	0.008	ND	0.0050 **±** 0.001	ND	**0.05∗**	0.029	0.06 **±** 0.03	0.06 **±** 0.05	0.13 **±** 0.02	**0.01** ^***β***^	ND	ND	ND	ND	**0.05∗**
*p,p'*-DDD	ND	0.005	0.004	0.006	**0.05∗**	0.039	0.057 **±** 0.009	0.046 **±** 0.004	0.24 **±** 0.04	**0.01** ^***β***^	ND	ND	ND	ND	**0.05∗**
*p,p'*-DDE	0.003	ND	ND	ND	**0.05∗**	0.582	0.003 **±** 0.0007	0.001 **±** 0.0002	0.0130 **±** 0.002	**0.01** ^***β***^	ND	ND	ND	ND	**0.05∗**
*p,p'*-DDT	ND	ND	0.015	ND	**0.05∗**	0.516	0.232 **±** 0.167	0.174 **±** 0.145	1.512 **±** 0.415	**0.01** ^***β***^	ND	ND	ND	ND	**0.05∗**
Cypermethrin	3.89 **±** 0.57	4.9 **±** 1.4	6.3 **±** 0.7	0.8 **±** 0.3	**0.01** ^***α***^	47.5 **±** 5.9	138.7 **±** 6.33	90.35 **±** 5.75	365.1 **±** 70.4	**0.01** ^***α***^ or **0.1∗**	2.99	3.2 **±** 0.2	2.87 **±** 0.58	2.8 **±** 1.2	**0.7** ^***α***^
Deltamethrin	0.015 **±** 0.004	0.022 **±** 0.002	0.005 **±** 0.003	0.012 **±** 0.005	**0.01** ^***α***^	0.85 **±** 0.29	0.61 **±** 0.25	0.46 **±** 0.16	1.19 **±** 0.38	**0.05** ^***α***^ or **0.06∗**	0.019 **±** 0.005	0.028 **±** 0.005	0.014 **±** 0.004	0.026 **±** 0.003	**2.0** ^***α***^ or **0.1**
Heptachlor	0.04 **±** 0.01	0.01 **±** 0.0003	0.06 **±** 0.007	0.07 **±** 0.009	**0.01** ^***β***^	0.18 **±** 0.008	0.42 **±** 0.15	0.18 **±** 0.12	0.75 **±** 0.24	**0.01** ^***β***^	0.013	0.006 **±** 0.001	0.01 **±** 0.002	0.25 **±** 0.009	**0.01∗**
*γ*-Chlordane	0.004 **±** 0.002	0.05 **±** 0.02	0.004 **±** 0.0002	0.004 **±** 0.001	**0.02** ^***α***^	0.005 **±** 0.0005	0.03 **±** 0.001	0.01 **±** 0.003	0.11 **±** 0.09	**0.02** ^***α***^	0.007	0.005 **±** 0.0009	0.004 **±** 0.002	0.005 **±** 0.0009	**0.02** ^***α***^ Or **0.01**
Dimethachlor	1.52 **±** 0.67	2.69 **±** 0.99	0.24 **±** 0.07	4.4 **±** 0.4	**0.01** ^***β***^	0.85 **±** 0.18	2.38 **±** 0.80	1.65 **±** 0.51	3.13 **±** 1.06	**0.01** ^***β***^	12.71	0.52 **±** 0.41	0.13 **±** 0.09	1.64 **±** 0.56	**0.01** ^***β***^
Lindane	0.02	0.04 **±** 0.006	0.05 **±** 0.01	0.06 **±** 0.01	**0.01** ^***α***^	0.14 **±** 0.006	0.37 **±** 0.04	0.21 **±** 0.06	0.81 **±** 0.24	**0.01** ^***α***^	0.005	0.03 **±** 0.009	0.008 **±** 0.002	0.03 **±** 0.007	**0.01** ^***α***^

*Note.* ND = not detected, MRL = maximum residue limit, *S*_1_ = mixed vegetable sample from Jimma town Merkato market, *S*_2_ = mixed vegetable sample from Jimma town Kochi market, *S*_3_ = mixed vegetable sample from Shebe market, *S*_4_ = mixed vegetable sample from Serbo market, *α* = Codex Alimentarius MRL value, *∗* = European Union MRL value, and *β* = recommended Default codex MRL for pesticides in food commodities without established maximum residue limit.

The article "Pesticide Residues and Effect of Household Processing in Commonly Consumed Vegetables in Jimma Zone, Southwest Ethiopia" was published in 2023. Journal: J Environ Public Health.

**Table 3:** Processing factor for the processes on pesticide residues in commonly consumed vegetables in Jimma Zone, southwest Ethiopia, 2021.

Processing factor (PF)													
Pesticides	Potato				Onion				Cabbage				
	Washing	Peeling	Boiling	Washing + peeling + boiling	Washing	Peeling	Boiling	Washing + peeling + boiling	Washing	Boiling	Washing + boiling using local method	Washing + boiling for 30 min	Washing + boiling for 1 hour
*o,p'*-DDT	0.31	0.35	0.43	0∗	0.62	**1.04**	0.38	0.11	0.36	0	0	0	0
*p,p'-*DDD	0.76	0.91	0.98	0.10∗∗	0.52	0.90	0.35	0.37	**1.23**	0.09∗∗	0.58	0.60	0.77
*p,p'-*DDE	0.59	0.17∗	0.91	0.05∗∗	0.92	0.39	**1.23**	0.19	**1.05**	0.26	0.60	0.68	0.85
*p,p'-*DDT	0.72	**1.58**	0.49	0.09	0.56	**1.18**	0.09	0.26	0	0	0	0.29	0.35

Cypermethrin	0.83	**4.74**	**1.13**	**2.97**	**11.05**	**9.35**	0.34	0.25	**1.44**	**2.00**	**2.13**	**4.78**	**4.94**
Deltamethrin	**2.02**	**8.51**	**2.25**	0	**1.42**	0.88	0.04	0.01	**1.75**	0.42	0.80	0.93	**1.37**

Heptachlor	**1.46**	**3.20**	**1.31**	0.05	0.67∗∗	0.54∗∗	0.08∗∗∗	0.03∗∗∗	**1.02**	0.40	0.95	0.51	0.99
*γ*-chlordane	0.63	0.75	0.68	0.03∗∗	0.70	**1.50**	0.56	0.27	**1.03**	0.28	0.79	0.85	**1.04**
Dimethachlor	**2.25**	**2.45**	**11.17**	0.71	0.42	0.42	0.05	0.05	0.72	0.28	0.27	0.73	0.55
Lindane	**1.56**	**2.33**	**2.40**	0.16	0.59	0.86	0.10	0.02	**1.06**	0.75	0.58	0.71	0.82

*Note.* PF < 1 (reduction factor) and PF > 1 (concentration factor), Bold indicated (concentrated), *∗* representing ANOVA with Tukey's post hoc test result with *P* < 0.05, *∗∗* for *P* < 0.01, and *∗∗∗* for *P* < 0.001

The article "Pesticide Residues and Effect of Household Processing in Commonly Consumed Vegetables in Jimma Zone, Southwest Ethiopia" was published in 2023. Journal: J Environ Public Health.

## Data Availability

The data set can be requested using the email adress of the crossponding author.
